The article "Hidradenitis suppurativa and cardiovascular diseases: A bidirectional Mendelian randomization study" was retracted in 2025. Reasons: compromised peer review; unreliable results or conclusions; concerns about the methods; concerns about the results or conclusions.

# Hidradenitis suppurativa and cardiovascular diseases: A bidirectional Mendelian randomization study

**DOI:** 10.1111/srt.13853

**Published:** 2024-07-17

**Authors:** Ping Zhou, Xin Jiang, Dan Wang

**Affiliations:** ^1^ Clinical Medical College Jiangxi University of Chinese Medicine Nanchang China; ^2^ Department of Dermatology Affiliated Hospital of Jiangxi University of Chinese Medicine Nanchang China

**Keywords:** cardiovascular diseases, causal relationship, gene, hidradenitis suppurativa, Mendelian randomization

## Abstract

**Background:**

Prior investigation has indicated a link between Hidradenitis suppurativa (HS) and cardiovascular diseases (CVDs), yet the causal relationship (CR) between these conditions remains unresolved.

**Methods:**

This investigation utilized bidirectional Mendelian randomization (MR) analysis to determine the CR between HS and CVDs. Genetic instruments for both conditions were sourced from genome‐wide association studies (GWAS). The GWAS summary data for CVD comprised coronary artery disease (CAD), myocardial infarction (MI), coronary atherosclerosis (CA), ischemic stroke (IS), and chronic heart failure (CHF). Four new approaches were added to the inverse variance weighted (IVW) method for the main analysis: weighted median, weighted MR‐Egger, simple mode, and weighted mode. The validity of the causal conclusions was verified by sensitivity tests that included leave‐one‐out analysis, heterogeneity, and pleiotropy.

**Results:**

HS and CAD (OR = 1.024; 95%CI: 1.002–1.046, *P* = 0.033), MI (OR = 1.001; 95%CI: 1.000–1.002, *P* = 0.033), and CA (OR = 1.001; 95%CI: 1.000–1.002, *P* = 0.022) were identified to have a positive CR, according to the IVW analysis. Conversely, no significant association was identified between HS and either IS or CHF. Furthermore, the bidirectional analysis indicated no reverse causation between these diseases.

**Conclusion:**

The findings of this study suggest a potential CR between HS and CAD, MI, and CA. Additional research is warranted to elucidate the biological mechanisms underlying these associations.

## 1 INTRODUCTION

A chronic inflammatory disease that affects the pilosebaceous unit, hidradenitis suppurativa (HS) is typified by recurrent inflammatory nodules, abscesses, draining skin tunnels, and scar formation. Usually, HS affects intertriginous areas like the groin, axillae, perianal region, perineum, and inframammary regions.^1^ The prevalence of HS ranges from less than 1% to 4%,^2^, ^3^ but it often results in pain, odor, discharge, and disfigurement, severely impacting patients’ psychological health and quality of life.^4^ Not all of the pathophysiology of HS is known; however, genetic predisposition, hormonal factors, follicular occlusion, follicular rupture, and associated immune responses appear to play crucial roles in its development and progression.^5^, ^6^, ^7^, ^8^

In recent years, several epidemiological studies have identified a strong correlation between HS and cardiovascular diseases (CVDs). A meta‐analysis evaluating the relationship between HS and cardiovascular risk factors found that, compared to a control group, individuals with HS had a markedly higher incidence of cardiovascular risk factors, including obesity, smoking history, diabetes, and metabolic syndrome.^9^ A study involving 5,964 patients with HS and 29,404 controls demonstrated that, after controlling for confounding factors such as obesity, smoking, and alcohol dependence, the risk of myocardial infarction (MI), ischemic stroke (IS), and cardiovascular‐related death was markedly increased in patients with HS.^10^ Research from the Hidradenitis Suppurativa Foundation in the United States and Canada also recommends screening patients with HS for CVDs, with a recommendation grade of IIB.^11^ Nonetheless, studies exploring the potential causal relationship (CR) and pathological mechanisms between HS and CVDs remain limited, necessitating further investigation.

The article "Hidradenitis suppurativa and cardiovascular diseases: A bidirectional Mendelian randomization study" was retracted in 2025. Reasons: compromised peer review; unreliable results or conclusions; concerns about the methods; concerns about the results or conclusions.

Observational studies traditionally test scientific hypotheses by comparing differences in outcome distributions between high and low exposure levels rather than through interventional exposure. However, reverse causality and other possible confounding variables could impact our findings. Using genetic variants as instrumental variables to determine the strength of the CR between exposure and result, Mendelian randomization (MR) is a genetic variable analysis technique that complies with Mendel's genetic law.^12^ MR employs genetic tools for instrumental variable (IV) analysis, and an individual's genotype is determined at conception and remains unchanged. Consequently, in contrast to retrospective research, MR lessens the interference of confounding factors and avoids reverse causality.^13^ In recent years, with the increasing sample size of genome‐wide association studies (GWAS) data, MR analysis has gained popularity as an effective method for inferring causality and has been widely applied. This analytical method has revealed CRs between HS and inflammatory bowel disease, gut microbiota, and atopic dermatitis.^14^, ^15^, ^16^ This study employs large‐scale GWAS summary data combined with MR analysis to identify the CR between HS and CVDs.

## 2 METHODOLOGIES AND MATERIALS

### 2.1 Study design

To explore the possible CR linking HS and CVDs, we employed MR analysis. In this approach, HS was considered the exposure variable, and single nucleotide polymorphisms (SNPs) strongly linked to HS were utilized as instrumental variables (IVs). The outcomes of interest encompassed five distinct CVD: coronary artery disease (CAD), myocardial infarction (MI), coronary atherosclerosis (CA), ischemic stroke (IS), and chronic heart failure (CHF). Subsequently, the roles of exposure and outcome data were reversed for a bidirectional analysis. This study adhered to three key assumptions: ① IVs should be highly correlated with exposure; ② IVs should not be influenced by variables that may potentially confuse the relationship between exposure and outcome; and ③ IVs should only affect the outcome as a direct result of exposure, without other pathways. The analytical procedure is depicted in Figure 1.

The article "Hidradenitis suppurativa and cardiovascular diseases: A bidirectional Mendelian randomization study" was retracted in 2025. Reasons: compromised peer review; unreliable results or conclusions; concerns about the methods; concerns about the results or conclusions.

**FIGURE 1:** Bidirectional two‐sample Mendelian randomization study workflow to comprehensively investigate the causal relationship between hidradenitis suppurativa and cardiovascular diseases. IVW, inverse variance weighted; SNPs single nucleotide polymorphisms.

### 2.2 Data sources

The HS GWA dataset was sourced from the latest and most comprehensive FinnGen R10 version, encompassing 1,070 cases and 394,105 controls of European ancestry. Data for CVDs were obtained from the IEU OpenGWAS project. No further ethical approval was needed because all of the data utilized in this analysis are publicly available. Table 1 presents comprehensive details about the datasets.

**TABLE 1:** Source of the GWAS data.

Traits	Data sources	Race	Sample size (cases/controls)	Datasets in the GWAS
HS	FinnGen	European	1,070/394,105	NA
CAD	CARD and UKB	European	122,733/424,528	ebi‐a‐GCST005195
MI	MRC‐IEU	European	10,616/452,317	ukb‐b‐15829
CA	Neale lab	European	14,334/346,860	ukb‐d‐I9_CORATHER
IS	MEASTROKE	European	7,193/406,111	ebi‐a‐GCST006910
CHF	EBI	European	14,262/471,898	ebi‐a‐GCST90018806

Abbreviations: CA, coronary atherosclerosis; CAD, coronary artery disease; CHF, chronic heart failure; GWAS, Genome‐Wide Association Studies; HS, hidradenitis suppurativa; IS, ischemic stroke; MI, myocardial infarction.

### 2.3 Instrument selection

To minimize potential bias from strong linkage disequilibrium between SNPs, rigorous screening criteria were applied: ① For HS as the exposure, SNPs with a significance level of *P* < 5 × 10^−6^ were utilized; for CVDs as the exposure, the threshold was *P* < 5 × 10^−8^. ② SNPs in linkage disequilibrium among the selected IVs were eliminated, with thresholds set at r^2^ < 0.001 and kb = 10000. ③ Relevant information for the selected IVs was retrieved from the GWAS data of the outcome, with allele alignment performed and palindromic sequences with intermediate allele frequencies removed. ④ Weak IVs were eliminated by calculating each SNP's F‐value; SNPs with an F‐value < 10 indicated weak IVs and were eliminated. The formula for calculating the F‐value is $F=\frac{R^{2}\times \left(N-K-1\right)}{K(1-R^{2})}\;$, where N is the sample size of the exposure, K is the number of SNPs; R^2^ is the proportion of variance explained by IVs; $R^{2}=\frac{2\times \beta^{2}\times \mathrm{EAF}\times \left(1-\mathrm{EAF}\right)}{2\times \beta^{2}\times \mathrm{EAF}\times \left(1-\mathrm{EAF}\right)+2\times SE^{2}\times N\times \mathrm{EAF}\times \left(1-\mathrm{EAF}\right)}\;$, β is the effect value, EAF is the effect allele frequency, and SE is the standard error of the β‐value.^17^, ^18^, ^19^ ⑤ To further minimize confounding, LDlink (https://ldlink.nih.gov/?tab = home) was used to exclude IVs associated with confounding factors.^20^

The article "Hidradenitis suppurativa and cardiovascular diseases: A bidirectional Mendelian randomization study" was retracted in 2025. Reasons: compromised peer review; unreliable results or conclusions; concerns about the methods; concerns about the results or conclusions.

### 2.4 MR analysis

This study included five different techniques: inverse variance weighted (IVW), MR‐Egger regression, weighted median, simple mode, and weighted mode, to ascertain CRs. The IVW method determines the weighted average of the effect sizes of all IVs during the analysis, providing relatively reliable results.^21^ Consequently, IVW results were selected as the primary indicator for assessing causal effects, while other methods were employed for supplementary evaluation. The outcomes are provided as 95% confidence intervals (CIs) and odds ratios (ORs), with *P* < 0.05 being employed to indicate statistical significance. The false discovery rate (FDR) for multiple testing was controlled utilizing the Benjamini‐Hochberg approach in light of the numerous MR studies that were performed.^22^ If *P* < FDR < 0.05, the two factors are considered markedly associated; if *P* < 0.05 < FDR, the association is deemed suggestive.^23^

### 2.5 Sensitivity analysis

Various techniques were employed to identify the presence of heterogeneity and pleiotropy. Cochran's Q statistic assessed heterogeneity among IVs in the IVW and MR‐Egger methods. Pleiotropy was identified utilizing the MR‐PRESSO test for the intercept term of the MR‐Egger regression; a *P* > 0.05 result revealed the lack of both pleiotropy and heterogeneity.^24^, ^25^, ^26^ Radial MR was used to identify and eliminate outliers.^27^ The robustness of the results was tested by progressively deleting each and every IV utilizing the leave‐one‐out strategy to identify the impact of specific SNPs on MR results.^28^

The analyses were primarily conducted utilizing R software (version 4.3.1) and the R packages TwoSampleMR (version 0.6.0), MR‐PRESSO (version 1.0), and RadialMR (version 1.1).

## 3 RESULTS

### 3.1 IVs

When utilizing HS as the exposure and CVD as the outcome, 16 SNPs were initially identified as IVs based on the established criteria. However, rs4713570 and rs7975017 were excluded due to their association with BMI, a known high‐risk factor for CVDs. For the reverse analysis, with CVDs as the exposure and HS as the outcome, the screened SNPs included 55 for CAD, 15 for MI, 27 for CA, four for IS, and six for CHF. The F‐statistics for each selected SNP exceeded 10, ranging from 21.071 to 595.219. Detailed information about the IVs is available in Table S1–S10.

The article "Hidradenitis suppurativa and cardiovascular diseases: A bidirectional Mendelian randomization study" was retracted in 2025. Reasons: compromised peer review; unreliable results or conclusions; concerns about the methods; concerns about the results or conclusions.

### 3.2 Causal effect of HS on CVDs

HS was linked to a higher risk of CAD, according to IVW analysis (OR = 1.024; 95% CI: 1.002 – 1.046, *P* = 0.033, *P*_FDR_ = 0.102). Similarly, the analysis revealed positive correlations between HS and MI (OR = 1.001; 95% CI: 1.000 – 1.002, *P* = 0.033, *P*_FDR_ = 0.163) and CA (OR = 1.001; 95% CI: 1.000 – 1.002, *P* = 0.022, *P*_FDR_ = 0.222). CAD incidence in patients with HS was 1.024‐fold higher than in the control group, and MI and CA incidences were 1.001‐fold higher. Conversely, no CR was identified between HS and IS (OR = 0.998; 95% CI: 0.950 – 1.049, *P* = 0.942, *P*_FDR_ = 0.942) or CHF (OR = 1.011; 95% CI: 0.993 – 1.029, *P* = 0.229, *P*_FDR_ = 0.382) (Figure 2A). The results are shown in Table S11.

**FIGURE 2:** (A) Using inverse variance weighted method to estimate the association between hidradenitis suppurativa and cardiovascular diseases; (B) Reverse Mendelian randomization estimate of the relationship between cardiovascular diseases and hidradenitis suppurativa. nSNP, number of single nucleotide polymorphisms; OR, odds ratio; CI, confidence interval.

### 3.3 Causal effect of CVDs on HS

Figure 2B illustrates that genetic susceptibility to CVDs does not have a CR with the risk of HS. The ORs and 95% CIs were as follows: CAD (OR = 0.861; 95% CI: 0.704 – 1.055, *P* = 0.149, *P*_FDR_ = 0.297); MI (OR = 0.051; 95% CI: 0.000 – 781.507, *P* = 0.545, *P*_FDR_ = 0.681); CA (OR = 0.019; 95% CI: 0.000 – 2.411, *P* = 0.109, *P*_FDR_ = 0.272); IS (OR = 0.938; 95% CI: 0.670 – 1.312, *P* = 0.708, *P*_FDR_ = 0.787); and CHF (OR = 0.267; 95% CI: 0.648 – 2.478, *P* = 0.490, *P*_FDR_ = 0.700). These findings suggest that genetic predisposition to CVDs does not markedly influence the development of HS. The results are shown in Table S12.

### 3.4 Sensitivity analysis of MR

The sensitivity analysis included tests for pleiotropy, heterogeneity, and leave‐one‐out analysis. In the MR‐Egger regression, there was no evidence of horizontal pleiotropy (intercept *P* > 0.05). Furthermore, both IVW and MR‐Egger analyses indicated no heterogeneity (Table 2). The leave‐one‐out analysis showed that the overall findings were not driven by any single SNP (Figure S1). The funnel plot (Figure S2) also visually confirmed the absence of heterogeneity in the analyzed data.

The article "Hidradenitis suppurativa and cardiovascular diseases: A bidirectional Mendelian randomization study" was retracted in 2025. Reasons: compromised peer review; unreliable results or conclusions; concerns about the methods; concerns about the results or conclusions.

**TABLE 2:** Sensitivity analysis of MR analyses.

		Pleiotropy test			Cochran's Q‐Test		
		MR‐Egger			MR‐Egger		
Exposure	Outcomes	Intercept	SE	*P*‐value	Q	Q‐pval	MR‐PRESSO
HS	CAD	−0.004	0.012	0.733	3.296	0.856	0.907
HS	MI	0.000	0.000	0.926	4.415	0.882	0.924
HS	CA	0.000	0.000	0.374	8.586	0.738	0.764
HS	IS	−0.022	0.018	0.250	11.341	0.415	0.408
HS	CHF	0.003	0.006	0.631	4.637	0.969	0.971
CAD	HS	−0.005	0.016	0.735	57.809	0.302	0.337
MI	HS	−0.048	0.044	0.298	7.495	0.875	0.825
CA	HS	0.027	0.029	0.366	19.335	0.781	0.792
IS	HS	−0.086	0.083	0.411	3.136	0.209	0.326
CHF	HS	−0.036	0.075	0.653	7.352	0.118	0.227

Abbreviations: CA, coronary atherosclerosis; CAD, coronary artery disease; CHF, chronic heart failure; HS, hidradenitis suppurativa; IS, ischemic stroke; MI, myocardial infarction.

## 4 DISCUSSION

This investigation is the initial attempt to utilize GWAS summary data to evaluate the CR between HS and CVDs. The analysis included five common CVDs: CAD, MI, CA, IS, and CHF. The MR analysis provided three key insights. Firstly, a suggestive positive CR was observed between HS and CAD, MI, and CA, indicating that HS may elevate the risk of developing these conditions. Secondly, no marked CR was identified between HS and either IS or CHF. Thirdly, the presence of CVDs did not correlate with an increased incidence of HS.

Prior observational research has looked into the connection between HS and CVDs.^29^, ^30^, ^31^, ^32^, ^33^ For instance, Reddy et al.^34^ found that, compared with non‐HS patients, those with HS had a 21% increased risk of MI after adjusting for relevant cardiovascular risk factors. A cohort study in Taiwan, which included 478 newly diagnosed patients with HS and 1,912 controls, also found that individuals with HS had a higher risk of suffering from CAD after adjusting for confounding factors (aHR: 2.722; 95% CI: 1.628–4.553; *P* < 0.001).^35^ Additionally, patients with HS exhibited an increased incidence of subclinical atherosclerosis compared to healthy controls.^36^, ^37^

HS is an immune‐mediated chronic inflammatory disease, and its inflammatory effects extend beyond the skin. The systemic inflammation resulting from the interaction of inflammatory factors and immune cells may contribute to an elevated cardiovascular risk.^38^ Blood tests in patients with HS have shown increased levels of cytokines IL‐1β and IL‐6, which can induce the liver to produce serum amyloid A, thereby increasing the risk of atherosclerosis.^39^ Research has also found that IL‐32 is overexpressed in both the lesional skin and serum of patients with HS.^40^ In addition to triggering pro‐inflammatory cytokines, including IL‐6, IL‐1β, and TNFα, IL‐32 can lead to endothelial dysfunction and reduce blood levels of high‐density lipoprotein, which increases the risk of developing CVD.^41^ It has been observed that HS patients with an inflammatory phenotype and higher C‐reactive protein levels are linked to an increased cardiovascular risk.^42^ Moreover, a new study has identified Trimethylamine N‐Oxide (TMAO) as a novel predictor of clinical severity in individuals with HS, showing a positive correlation with disease severity.^43^ Interestingly, TMAO can bind to protein kinase R‐like endoplasmic reticulum kinase to induce the transcription factor FoxO1, promoting cardiac metabolic diseases.^44^ Long‐term elevation of TMAO levels is linked to a higher risk of CVD.^45^ Given these findings, it is hypothesized that inflammatory factors may mediate the CR between HS and cardiovascular risk.

The article "Hidradenitis suppurativa and cardiovascular diseases: A bidirectional Mendelian randomization study" was retracted in 2025. Reasons: compromised peer review; unreliable results or conclusions; concerns about the methods; concerns about the results or conclusions.

The merit of this study is its extensive MR analysis that reduces confounding factor interference by using data from public databases. The findings’ dependability is further supported by the sensitivity and heterogeneity analysis. However, several limitations must be acknowledged. First, the data sources are predominantly from the European population; therefore, attention should be paid to extrapolating the results to other ethnicities. Second, while the results were adjusted for multiple testing, the outcomes tend to be more conservative due to the relatively modest impact of HS on these diseases. Larger sample numbers or more reliable genetic instrumental factors could be needed for validation in further research. Third, the absence of detailed demographic information and clinical characteristics of the participants precluded subgroup analyses. Lastly, this study did not investigate the potential mechanistic pathways that may mediate the observed associations. Further investigation is warranted to identify the relationship between HS, CVDs, and inflammatory factors, as shared inflammatory factors between the two conditions may become critical therapeutic targets for preventing these diseases and their complications.

## 5 CONCLUSION

This study elucidated the genetic impact of HS on common CVDs. It identified a potential CR between HS and CAD, MI, and CA, indicating a possible link between HS and these CVDs. Clinicians treating patients with HS should consider not only the management of skin symptoms but also be vigilant about this potential risk to mitigate complications and reduce mortality.

## CONFLICT OF INTEREST STATEMENT

The authors declare no conflicts of interest.

The article "Hidradenitis suppurativa and cardiovascular diseases: A bidirectional Mendelian randomization study" was retracted in 2025. Reasons: compromised peer review; unreliable results or conclusions; concerns about the methods; concerns about the results or conclusions.

## ETHICS STATEMENT

Not applicable.

## Supporting information

Supplementary Information

Supplementary Information

## Data Availability

The data for this research were sourced from public databases. FinnGen provides access to the GWAS summary data for HS at https://r10.finngen.fi/. The IEU OpenGWAS database, accessible at https://gwas.mrcieu.ac.uk/, contains the GWAS summary data for the five CVDs.
